This article has been retracted.

# Research on the Impact of Regional Economy on Industrial Development from the Perspective of Big Data

**DOI:** 10.1155/2021/5990655

**Published:** 2021-12-14

**Authors:** Lu Zhang, Dong Zhao, Siheng Li, Han Xiao, Jianjun Bu, Marvin White

**Affiliations:** ^1^School of Economics & Management, Yancheng Institute of University, Yancheng, 224007 Jiangsu, China; ^2^Southern Chongqing Regional Company of Country Garden Holdings, China Resources Building, Xiejiawan Street, Jiulongpo District, 400050 Chongqing, China; ^3^University of International Business and Economics, Institute of Education and Economy Research, Beijing, 100029 Beijing, China; ^4^Suzhou University, China; ^5^Shanxi University, China; ^6^Department of Information Engineering, Southern University and A&M College, Louisiana, USA

## Abstract

In order to study the driving force of China's rapid economic development in the past ten years, the study takes Guizhou, Yunnan, and Guangxi as a case study, focusing on the big data assets exchange (GBDEx) and Beibu Gulf Economic Zone, and discusses the impact of Internet plus economic and government data and the big data system on regional economy. Finally, it is believed that the Internet and big data fully avoid the disadvantages of traffic distance between the western region and the eastern region, make full and efficient cooperation between enterprises and institutions in the central and western regions and Chinese and foreign economic entities, and strengthen the control of economic behavior from the big data level with the support of the service-oriented government. The information entropy output from the Internet big data system has led to a significant entropy reduction process in China's economic environment and a more orderly economic system, which is also an important reason for the rapid development of China's economy.

## 1. Introduction

Since the 17th Congress of the Communist Party of China, a number of regional economic development strategies have been established throughout China, including the Xiong'an Start-up Area centered on Beijing and its expanded Bohai Sea Economic Zone, the Guangdong-Hong Kong-Marco Greater Bay Area centered on Guangzhou and Shenzhen and its expanded Beibu Gulf Economic Zone and Hainan Free Trade Zone, and the Yangtze River Delta Economic Zone centered on Shanghai, Zhongyuan Economic Zone centered on Zhengzhou and Kaifeng, Sichuan Chongqing Economic Zone centered on Chongqing, and Internet finance pilot development zone centered on Guizhou. The research takes the pull model of Guizhou Internet finance to the regional economy as the key technology to deeply explore relevant topics [1]. The Yangtze River Delta is one of the regions with the most active economic development, the highest degree of openness, and the strongest innovation ability in China. It plays an important strategic role in the overall situation of national modernization and all-round opening-up pattern. Promoting the integrated development of the Yangtze River Delta, enhancing the innovation and competitiveness of the Yangtze River Delta, and improving the degree of economic agglomeration, regional connectivity, and policy coordination efficiency are of great significance to leading the country's high-quality development and building a modern economic system.

Early big data is a concept of computer network technology. After the Internet plus economic model is put forward and implemented, big data has become a sociological concept, which is related to data security, data application, and data assets. GBDEx, also known as Guiyang big data asset exchange, is the third securitization asset trading platform established after Shenzhen Stock Exchange and Shanghai Stock Exchange under the promotion of the Chinese government [2]. The big data resources owned by enterprises can only be classified into the financial asset system from intangible assets in the early stage, and more enterprises only treat them as projects under construction, which leads to low profits and low taxes payable by science and technology enterprises on the one hand, and financing difficulties for science and technology enterprises on the other hand [3]. The specific performance of microenterprises and regional economy under the financial strategy of big data assets will be discussed below. Big data is defined as a data set with a large scale that greatly exceeds the capabilities of traditional database software tools in terms of acquisition, storage, management, and analysis. It has four characteristics: massive data scale, rapid data flow, diverse data types, and low-value density. The strategic significance of big data technology lies not in mastering huge data information, but in the professional processing of these meaningful data. In other words, if big data is compared to an industry, the key to the profitability of this industry lies in improving the “processing capacity” of data and realizing the “value-added” of data through “processing.”

## 2. Detailed Explanation of China's Western Development Strategy

Beibu Gulf Economic Zone, with ASEAN foreign trade as the main development driving force, is driven by GBDEx, Hainan free trade zone, and Yangtze River Delta economic zone. While realizing ASEAN external circulation, it drives the internal circulation mode of local economy and realizes the double circulation of China's economy [4]. The above architecture is shown in Figure 1: the main task of Beibu Gulf Economic Zone is to build it into a logistics base, trade base, processing, and manufacturing base and Information Exchange Center for China ASEAN open cooperation. The functional orientation of the Beibu Gulf Economic Zone is based on the Beibu Gulf, serving the “three South” (southwest, South China and Central South), connecting East, West and East, and facing Southeast Asia, give full play to the role of an important channel, exchange bridge and cooperation platform connecting multiple regions, promote development and construction through opening and cooperation, and strive to build a logistics base, trade base, and processing and manufacturing base and information exchange center.

In Figure 1, under the guidance of the basic development concept of getting rich first and driving getting rich later, there are three ways to support the Beibu Gulf Economic Zone [5]: (1) the core city of one belt, one road of the western development strategy, is Chongqing. Chongqing city was reestablished in 1997. It is the east bridgehead of Chongqing-Sinkiang-Europe International Railway. The railway is Kazakhstan, Russia, Belarus, Poland, and Germany. It is an important link between China and Europe. At the same time, it will stimulate the development of brewing industry, computer hardware manufacturing industry, high-tech development, and higher education system in the central and western regions. (2) Guiyang Internet financial development center undertakes the legalization mission of internet finance naturally formed in the economic system with Chinese characteristics. It is the core pilot area of China's financial system reform. One of the core tasks of the pilot is to securitize enterprise big data assets and realize online bargaining under the supervision of multiple departments. In addition, Internet financing business is also actively exploring the legalization process in Guiyang development zone. (3) Hainan free trade zone is a large pilot free trade zone with the largest area and the second-largest economic volume in the Far East. In the future, its economic volume may reach the first in the Far East. In addition, small port free trade bonded zones such as Shanghai free trade zone and Chongqing Free Trade Zone produce the pulling effect of economic external circulation at the same time. Beibu Gulf Economic Zone, centered on Beihai City and Fangchenggang City, Guangxi Province, is designed to promote international trade between China and ASEAN. However, under the dual economic cycle, its essential purpose is to fully stimulate the internal economic cycle volume of southern Guangxi and drive the all-round economic development of southwest provinces and autonomous regions such as western Guangdong, Guangxi, Yunnan, and Guizhou.

Taking Beibu Gulf Economic Zone as an example, regardless of the supporting role of other economic zones and economic development promotion facilities [6], the logical structure relationship between its internal economic entities is shown in Figure 2. The development goal of Beibu Gulf Economic Zone is to build it into an important coastal economic growth area in China after 10 to 15 years of efforts and take the lead in realizing the goal of building a well-off society in an all-round way in the western region.

In Figure 2, there are six core economic modules: (1) the core function of Beibu Gulf Economic Zone is a tariff free and low enterprise income tax trade logistics system based on Beihai wharf and Fangchenggang wharf. Among them, among the 28 berths of Fangcheng Port Wharf, the maximum can accommodate 200000 tons of ships, among the 31 berths of Beihai wharf, the maximum can accommodate 70000 tons of ships, and 150000 ton berths are under planning and construction. That is, Fangcheng port terminal mainly undertakes the task of ocean transportation logistics, and Beihai terminal mainly undertakes the task of offshore transportation logistics in ASEAN and the Western Pacific. (2) Before the establishment of Beibu Gulf Economic Zone, Beibu Gulf was the core producing area of China's oil and gas, and the oil industry was its original industrial foundation in the early stage of the establishment of Beibu Gulf Economic Zone. (3) The international trade function between China and ASEAN is the initial function in the preparation for the establishment of the Beibu Gulf Economic Zone. After the comprehensive construction of the two port cities, the trade function between China and other maritime neighbors has gradually joined. Moreover, Chongqing Sinkiang Europe International Railway extends southward from Chongqing, enters Guangxi through Guizhou, connects with the two major ports, and fully integrates the trade functions between China and Europe. (4) Guangxi autonomous region is a minority autonomous region, and the ecological characteristic agriculture and tourism industry with national characteristics account for a large proportion of the local economy. Tea, flowers, tropical and subtropical fruits, and vegetables, as well as the planting environment of three crops a year in some local areas, make local agriculture overcome the difficulties of many mountains and valleys and become an important economic element. (5) After the establishment of Beibu Gulf Economic Zone, affected by local investment policies, including full tariff exemption, minimum 9% enterprise income tax, green channel for industrial land approval, etc., it has attracted a large number of computer hardware manufacturing and other related enterprises, especially cooperating with storage hardware enterprises in Southeast Asia, fully combine Chinese highly educated and high-quality workers with ASEAN computer storage hardware production capacity. At the same time, China's key industries in recent years, such as chip manufacturing, flexible screen manufacturing, and mobile phone parts manufacturing, are also developing in an all-round way in the Beibu Gulf Economic Zone. (6) The Beibu Gulf Economic Zone supports scientific and technological R & D institutions much more than scientific and technological manufacturing enterprises. Therefore, many well-known higher education institutions at home and abroad, including many 211 Project universities, set up key laboratories and postdoctoral workstations in the Beibu Gulf Economic Zone, which are fully integrated with local scientific and technological manufacturing enterprises and ecological agriculture development enterprises, quickly and efficiently realize the transformation of industry, university, and research. The scientific research projects less reported by the media also include China's breeding project and animal husbandry optimization project comprehensively promoted by the Chinese government's no. 1 document over the years, and a large number of scientific research tasks undertaken by the science and technology development project of Beibu Gulf Economic Zone.

The state strongly supports the opening-up and development of Beibu Gulf Economic Zone and clearly gives policy support in five aspects: policy support for comprehensive supporting reform, and the State supports the promotion of comprehensive supporting reforms such as administrative system, market system, and land management system. The state provides policy support for the layout of major projects in terms of relevant planning, layout of major projects and project approval, approval, and filing. In terms of policy support for the bonded logistics system, the State supports the Beibu Gulf Economic Zone to set up bonded port areas, comprehensive bonded zones, and bonded logistics centers in qualified areas, and expand the bonded logistics function of export processing zones. In terms of policy support for financial reform, the State supports the establishment of local banks in the Beibu Gulf region, explores the establishment of industrial investment funds and venture capital enterprises, expands the issuance scale of corporate bonds, and supports qualified enterprises to issue corporate bonds. In terms of policy support for opening up and cooperation, the State supports the Beibu Gulf Economic Zone to play an exemplary role in opening up and cooperation, promote Pan Beibu Gulf Economic Cooperation to become a new subregional cooperation under the China ASEAN cooperation framework, establish and improve the opening and cooperation mechanism, and accelerate the implementation of cooperation projects.

## 3. Specific Performance of Southwest Regional Economy

China's western development strategy has been implemented for more than ten years. In the past ten years, the regional development speed represented by Guangxi Autonomous Region, Yunnan, and Guizhou is much higher than the national average and also higher than that of early development provinces such as Beijing, Shanghai, and Guangdong [7]. The development data are shown in Table 1.

The development of the west is related to the overall situation of China's modernization: the difficulty of China's modernization lies not in the East, but in the West; the ultimate goal of China's modernization may also be in the western region. Therefore, developing the west is a development strategy and strategic task that must be adhered to for a long time. The whole 21st century should pay attention to the development of the West. China's traditional industrialization process has not been completed, the modernization process has not started long, and the fundamental transformation of the economic system and economic growth mode has not been completed. The development of the whole country is unbalanced, and so is the development of the western region: the problem of regional gap is basically the problem of urban-rural gap.

A senior researcher of China's Ministry of industry and information technology pointed out that the essence of the Internet economy has nothing to do with the traditional IT industry. Its essence lies in the infinite fine division of labor and highly close cooperation of the industry. That is, China's Internet economy is not based on the data exchange of electronic equipment, but the deep, interactive, and reliable cooperation between natural persons and enterprise legal persons. Transforming the data communication service between traditional electronic devices into data sharing between natural persons and corporate legal persons is the manifestation of China's Internet plus economy. In Table 1 above, there are two main reasons for the rapid economic development in Western China: (1) national policies are fully inclined to the western region, including tax policies, land policies, and financial policies. The policy environment of the western region is significantly better than that of the early developed eastern coastal areas, and the people also have the investment orientation of “policy highland” and “tax lowland.” (2) Under the guidance of the concept of social development with Chinese characteristics, the enterprise legal persons and natural persons in the first rich areas do not actively support the latter rich areas, but form a social public identity and interest guidance channel for investment and development in the central and western regions. Under the self-driving force of social game theory and Nash equilibrium, the investment from the first rich areas to the latter rich areas in the central and western regions becomes the optimal game result. Solving the problems of data sharing and information public opinion dissemination in the first rich areas and the second rich areas has become the key technology of the above two development drivers. When college graduates participate in the western service plan and work at the grass-roots level, the municipal and county finance will give them certain living subsidies; working in rural areas; students can be arranged to hold corresponding positions in the village Party branch and village committee through legal procedures; the length of service shall be calculated during the service period, and the party League relationship shall be transferred to the service unit. Volunteers who have passed the examination after the expiration of their service will be given extra points when applying for graduate students. Upon the expiration of the service period, the volunteers shall be identified and stored in their own files; those who pass the examination will be issued with certificates as proof of volunteer service experience, employment, and entrepreneurship.

Although the Internet plus economic mode is not aimed at data communication between electronic devices, the traditional Internet-based facilities based on electronic hardware have direct support for the Internet plus economy [8], as shown in Figure 3.

In Figure 3, manufacturing enterprises that adapt to the Internet plus economic environment have six Internet functions [9]: (1) Internet administration and finance: under the government affairs 4.0 mode, all enterprises and government management departments can exchange data through the Internet interface, including the submission and approval of various reports in the field of administration, the online submission of various financial statements and tax statements, tax withholding, etc. (2) Internet enterprise collaboration: while Internet enterprises establish Internet data interaction interfaces with relevant government departments, Internet enterprises also establish interaction and collaboration interfaces, including data sharing between enterprises, online signing, etc. Financial services, insurance services, hydropower and energy services, property services, consulting services, etc. can achieve full collaboration without travel negotiation through the collaborative cooperation Internet interface between enterprises. (3) Internet personnel system: high-quality migrant workers projects led by local governments, service platforms for various labor dispatch enterprises and professional managers, and Internet service platforms for highly educated and professional technicians can form synergy with enterprises through Internet channels. Internet enterprises can directly obtain high-quality workers, managers, technicians, and other teams by accepting the services of relevant internet platforms. (4) Cloud manufacturing system: the cloud manufacturing concept originally proposed by the B2B Internet platform is an Internet collaboration mode for enterprises to fully share means of production, including workshops, equipment, processing technology, technical worker team, processing qualification, etc. For example, for orders in the Yangtze River Delta, Pearl River Delta, and other regions, you can find nationwide processing sites on this platform to realize workshop-free and approval-free processing and production. Because of the low price of industrial land and labor, the western region can seek cloud manufacturing orders through the platform. (5) Internet R & D system: scientific research projects in Colleges and universities need to form benefits through the transformation of industry, university, and research, and scientific research achievements also need to serve the society through the transformation of industry, university, and research. Under the Internet R & D mechanism, all signing and interaction processes can be realized through Internet big data. (6) Internet office system: an important feature of Internet enterprises is that they have multiple office locations. For example, for enterprises registered in the western region, their headquarters are generally still in large coastal cities in the East. Therefore, internal departments of enterprises also need to realize coordination through the Internet. At the same time, the human resource cost of more high-quality talents is high, and enterprises generally share high-quality talents. Therefore, some high-quality talents will also form independent studios and form Internet Office coordination channels between their cooperative enterprises. Cloud manufacturing is a new concept developed based on the concept of “manufacturing as a service” and the idea of cloud computing. Cloud manufacturing is a cross integration product of advanced information technology, manufacturing technology, and emerging Internet of things technology. It is the embodiment of the concept of manufacturing as a service. Adopt the cutting-edge concept of contemporary information technology, including cloud computing, to support the manufacturing industry to provide products with high value-added, low-cost, and global manufacturing services under a wide range of network resources.

## 4. Political and Economic Principles of China's Western Development

Even if Chinese mainland economy lagged far behind some parts of China, including Japan, Korea, Singapore, India, and Thailand, China's economic volume and political and economic management level far exceeded that of China, even the economic level of China's Hongkong, Taiwan, and Macao regions was higher than that of mainland China only ten years ago. In 10 years, China has surpassed more than 10 countries and regions and developed into the world's second largest economy and the world's largest industrial economy, which contains many innovations in political economy. The Internet plus economic model is the key [10]. The Internet plus basic connotation is an upgraded version of integration of information and industrialization. Taking the Internet as the core feature of the current information development, it is extracted and integrated with industry, commerce, and finance. The key is innovation. Only innovation can make this + truly valuable and meaningful. Internet plus. It is considered to be a new form and business form of Internet development under Innovation 2.0, and the evolution of a new form of economic and social development driven by Innovation 2.0 of knowledge society.

### 4.1. Theory of Government Enterprise Relationship from the Perspective of Ecological Economics

From 1956 to 1978 (one way of saying to 1995), the Chinese government's supervision of enterprises belongs to a strong supervision mechanism. Various public utilities were established under the government to carry out administrative management of relevant enterprises. After 1995, various public utilities were transformed into state-owned group companies. In this context, even today, various administrative affairs of enterprises still need to submit reports to the government regulatory authorities and get administrative approval. This regulatory model was once criticized by western economists, but practice has proved that China has formed an enterprise survival ecology with Chinese characteristics under this regulatory model.

The new government enterprise cooperation mode with Chinese characteristics formed under the condition of government affairs 4.0 is fully benefited from government affairs big data, and its era characteristics are shown in Figure 4.

In Figure 4, service-oriented government is a government organization mode corresponding to minimizing government in western public service theory, and it is also a specific practice of government functions with Chinese characteristics. Under the government affairs 4.0 system, the government assists the data interaction between enterprises and various legal entities and promotes their cooperation and coordination by managing economic big data. This is the key theoretical basis of political economy for the rapid development of China's economy in the past decade. Therefore, in China, economic big data is the technical expression of social economy, and the Internet is the effective management of economic big data. Under the promotion of the Internet plus economic mode, the western regions with relatively backward development and the early Eastern regions developed into the process of full integration of big data. Ultimately, the process of economic development in the western region can be effectively assisted by the eastern region, which eventually leads to the development speed of the western region far beyond that of the East (see Table 1 above). Based on cloud computing technology, some Internet enterprises have created a unified software service platform for intelligent products, provided unified software services and technical support for intelligent hardware devices produced by different manufacturers, optimized the user experience, realized the interconnection of various products, and generated collaborative value.

### 4.2. The Information Entropy to Social Balance

In 1948, the concept of information entropy was put forward by the western philosopher C. E. Shannon. It is a fusion concept of sociology and thermodynamics. The basic philosophical world outlook theory of this theory holds that social phenomena belong to natural phenomena, so they should be affected by the mathematical laws of nature. Its mathematical expression is shown in the following formulas:

(1) $$\begin{array}{c} f\left(P\right)=\log\frac{1}{p}=-\log P,\\ H\left(U\right)=E\left|-\log p_{i}\right|=-\overset{n}{\underset{i=1}{\sum }}p_{i}\log p_{i}, \end{array}$$

where *P* is the probability statistical result under specific mode; *U* is the constrained independent variable of probability statistics, which can be summarized as *U*{*u*_1_, *u*_2_, *Λ*, *u*_*i*_}; *p*_*i*_ is the *i*th probability statistical result under the condition of constrained independent variable; *H* is information entropy.

In the theory of information entropy, although the entropy of the basic rules of the universe only increases without decreasing, information entropy is the only way to provide inverse entropy to closed systems and lead to entropy reduction. The information resources provided by Internet big data contribute to the social structure, cause the ordering of local social forms, and promote the rapid development of social economy.

### 4.3. Economic Development Model under the Condition of Social Self-Drive

Comparing 2010 before the implementation of the Internet economic model with 2020 after the implementation of the Internet economic model, the proportion of GDP and growth rate of the three major industries in Guangxi Province and Yunnan Province are shown in Table 2.

In Table 2, China's economic statistics divides agricultural industry into primary industry, industry and mining industry into secondary industry, and finance and service industry into tertiary industry. In the three economic regions of Guangxi, Yunnan, and Guizhou investigated in this study, there are significant differences in the growth of the three industries in recent 10 years. The primary industry in Guizhou Province has developed rapidly and affected by the rapid growth of logistics service industry, the tertiary industry in the three provinces has increased in a large proportion. However, although Guangxi Province is the core province of Beibu Gulf Economic Zone, the development speed of the three major industries is not as fast as that of Guizhou Province, which comprehensively promotes the Internet economic model. It can be seen that Guizhou Province is the core driving force of the western development, while Guangxi province still needs to further explore the regional economy. In the future, the Internet plus economic mode will be the core and main structure of China's economic model with Chinese characteristics. Regional economic management departments and decision-makers should fully understand the economic and sociological attributes of the Internet, give full play to the management and control ability of government departments over the Internet and big data, and make the regional economy develop rapidly with the full help of Internet big data.

## 5. Summary

The regional economic development in Western China has been significantly promoted by the Internet economy and big data management system. Guizhou Province, where Guiyang big data exchange is located, has a more rapid development than the surrounding Guangxi Autonomous Region and Yunnan Province, and Guangxi Autonomous Region, Guizhou Province, and Yunnan Province have a faster development speed than Guangdong Province, Shanghai Municipality, and Beijing Municipality in the East. The principle of Internet and big data promoting the development of the western region is that they fully integrate the national economic entities, solve the traffic distance between the western region and the eastern region, but give full play to the low development cost of the western region. China's one belt, one road cooperation between Xinjiang and the Middle East and Iran, and the Sino European cooperation model with Europe are also included in the study. Due to China's special geography and landform, most of the land transportation ports of neighboring countries are concentrated in the West. The important way of western development is to promote domestic economic cooperation and comprehensively develop international trade.

## Figures and Tables

**Figure 1:** Guiyang Internet finance, Hainan free trade zone, and western development strategy (southwest part).

**Figure 2:** Basic economic structure of Beibu Gulf Economic Zone.

**Figure 3:** Schematic diagram of enterprise operating environment under Internet plus economic mode.

**Figure 4:** Internet big data structure of service-oriented government participating in enterprise ecology.

**Table 1:** Economic development data of central and Western China in recent ten years (based on GDP) (unit: USD 100 million) (data source: National Bureau of Statistics).

Region	2020	2019	2010	Year-to-year growth	Ten-year growth
Guangxi	3408.7	3267.3	1215.9	4.33%	168.71%
Yunnan	3772.6	3572.9	950.5	5.59%	275.90%
Guizhou	2742.5	2579.9	563.5	6.30%	357.87%
Beijing	5554.2	5441.7	1764.5	2.07%	208.40%
Shanghai	5953.9	5844.2	2206.9	1.88%	164.82%
Guangdong	17040.1	16564.8	5811.6	2.87%	185.03%
Nationwide	156307.7	152440.8	61771.2	2.54%	146.78%

**Table 2:** Changes in the proportion of economic components (data source: Statistics Bureau).

Comparison items	Industrial gradient	Guangxi	Yunnan	Guizhou
2020	Agricultural industry	3555.82	3598.91	2539.88
	Industrial and mining industry	7108.49	8287.54	6211.62
	Financial and service industry	11492.38	12635.45	9075.07

2010	Agricultural industry	1675.06	1108.4	625.03
	Industrial and mining industry	4511.68	3223.5	1800.06
	Financial and service industry	3383.1	2892.3	2177.07

Ten-year growth	Agricultural industry	112.28%	224.69%	306.36%
	Industrial and mining industry	57.56%	157.10%	245.08%
	Financial and service industry	239.70%	336.87%	316.85%

## Data Availability

The data underlying the results presented in the study are available within the manuscript.
